The article "The scourge of substandard and falsified medical products gets worse with COVID-19 pandemic" was published in 2020. Journal: Pan Afr Med J.

# The scourge of substandard and falsified medical products gets worse with COVID-19 pandemic

**DOI:** 10.11604/pamj.2020.37.344.26322

**Published:** 2020-12-15

**Authors:** Fisseha Shiferie, Eden Kassa

**Affiliations:** 1 Addis Continental Institute of Public Health, Addis Ababa, Ethiopia,; 2 Defense Health Science College, Debre Zeit, Ethiopia

**Keywords:** Substandard, falsified, COVID-19, regulatory body

## Abstract

Although health professionals, communities, governments and global institutions work closely to halt the spread of COVID-19 and mitigate its societal impact, COVID-19 remains a challenge to many countries around the world. In addition to its direct health, economic and social consequences, the pandemic has also resulted in unforeseen consequences in Africa especially in East African countries. COVID-19 might increase the demand and consumption of Substandard and Falsified (SF) medical products in three major ways. The first way is due to the inability of vulnerable segment of the population to access healthcare services as they used to do before. The second way people get exposed to SF medical products is due to fear of being quarantined, isolated and traced. Yet another way is related to import permits for medical products. Concerned regulatory bodies shall intervene aggressively in ensuring the safety, quality and effectiveness of medical products before we face a parallel pandemic from SF medical products.

## Commentary

### Introduction

On 31^st^ December 2019, the World Health Organization (WHO) was informed of a cluster of cases of pneumonia of unknown cause, first of which reported on 09^th^ December 2019, detected in Wuhan City, Hubei Province of China. The severe acute respiratory syndrome coronavirus 2 (SARS-CoV-2) was identified as the causative virus by Chinese authorities on 7^th^ January, with evidence of human-to-human transmission by 20^th^ January. On 30^th^ January 2020, the outbreak was declared a Public Health Emergency of International Concern (PHEIC) and a pandemic on March 11^th^, 2020 [1]. As health professionals, communities, governments and global institutions work closely to halt the spread of COVID-19 and mitigate its societal impact, COVID-19 remains a challenge to many countries around the world [2]. As of 12^th^ October 2020, there are over thirty-seven million confirmed cases and over 1,000,000 have died from the virus worldwide. In Africa, the total number of confirmed cases is over 1,500,000 while those that have died from the virus are over 38,000 [3]. Most studies have explored the health, economic and social consequences resulted directly from COVID-19. However, the pandemic has also resulted in unforeseen consequences in Africa especially in East African countries. In this study, we focused on the effect of the pandemic on the consumption of substandard and falsified medical products.

The article "The scourge of substandard and falsified medical products gets worse with COVID-19 pandemic" was published in 2020. Journal: Pan Afr Med J.

### Analysis and discussion

The United Nations has declared access to safe, effective, quality, and affordable essential medicines to be one of the Sustainable Development Goals (SDGs) in their 2030 Agenda. Still, substandard and falsified (SF) medical products represent a serious problem for public health, especially in Africa, South-East Asia and Latin America [4]. Substandard medical products can be defined as authorized medical products that fail to meet either their quality standards or specification, or both, according to the World Health Organization (WHO) and may result through poor manufacturing, shipping or storage conditions, or when the drug is sold beyond the expiration date. Falsified medicines, on the other hand, are medical products that deliberately misrepresent their identity, composition or source [5].

Risks posed by SF medical products can be broadly categorized as health and economic consequences. Health-related consequences of SF medicines include, but are not limited to, risks of morbidity and mortality (resulting from either treatment failure or adverse drug reactions), drug resistance and erosion of patients´ trust on the healthcare system, healthcare providers and genuine drug manufacturers. By the same token, its economic consequences include increased costs for patients and governments, reduced economic productivity and poverty [6-9].

COVID-19 and substandard and falsified medicines share one thing in common: both are global public health threats. However, COVID-19 and SF products are different in many fundamental ways. Obviously, COVID-19 is a disease, but the latter is not. While COVID-19 is affecting both developed and developing nations invariably, the profound impact of SF medical products is more pronounced in low- and middle-income countries. It is estimated that 10% of medical products in developing countries are SF, according to WHO. Due to the current increased demand for medicines, vaccines and reagents following the pandemic, the prevalence of SF will increase.

COVID-19 might increase the demand and consumption of SF medical products in three major ways. The first way is due to the inability of vulnerable segment of the population such as pregnant women, individuals working in the informal sector, and patients with comorbidities to access healthcare services. As a means to curb the transmission of the virus and prevent its devastating consequences, governments declared state of emergency (SOE). As part of the SOE, a stay-at-home (SAH) or work-from-home (WFH) measures were issued. Businesses, schools and Universities are closed. Transportation tariff has doubled as a compensation for the 50pc reduction of passenger loads. With the stay-at-home orders and increased tariffs, millions of individuals might face unprecedented difficulties to access healthcare services. Essential medicines are one of them. It is during this time that these people get exposed to SF medical products.

The article "The scourge of substandard and falsified medical products gets worse with COVID-19 pandemic" was published in 2020. Journal: Pan Afr Med J.

The inevitable consequences of SF medical products are not only limited to people working in the informal sector. It also affects the other vulnerable segments of the population such as people living with HIV/AIDS (PLWHA), patients with comorbidities, communities living in malaria-endemic settings, pregnant women and people under treatment for tuberculosis. It is also quite unavoidable that the pandemic would take attention away from routine healthcare services. Take pregnant women, who are expected to visit health facilities as frequently as possible. With the pandemic taking the air out of the attention from other health services, women´s and their babies´ health will definitely be at high risk. This will open the door for ill-intended SF dealers to easily distribute their products. The risk posed to the remaining vulnerable segment of the population is no different.

The other way for people to get exposed to SF medical products is due to fear of being quarantined, isolated and traced. Quarantine of suspected cases and isolation of COVID-19 patients and contact tracing are the strategies being implemented to contain the spread of the virus. The acceptability of these measures by the community has not been encouraging though. Fear of being quarantined and isolated might force people to use whatever is available in the market as a substitute for visiting healthcare facilities. In this regard, the chances of accessing SF medical products are very high. Yet another way is related to import permits for medical products. Since the first case (index) was reported in most countries in East Africa, an overwhelming number of applications from medicine and medical supplies importers are being filed in their respective drug regulatory authorities. Given the magnitude of the problem COVID-19 has brought, governments have given priorities and incentives to importers that have submitted applications to import COVID-19 related medical supplies such as face masks, hand sanitizers and gloves. This is a good and timely decision in terms of filling the personal protective equipment (PPE) shortage we are facing.

However, in East African countries where there is an already existing shortage of essential medicines, the tight window through which these products are allowed to come in is tantamount to “adding fuel to the fire”. It complicates the problem and will be a good recipe for dealers of SF medical products to easily penetrate the market. The threat from SF medical products will continue even post COVID-19 era unless strict measures are taken by the government. Genuine importers, healthcare providers and end-users should be vigilant in the war against SF medical product dealers. One way of overcoming such threats, especially for consumers, is by following certain general guidelines that can go a long way in combating the flood of SF medicines products. People need to look at the packaging, spelling mistakes and grammatical errors before purchasing these items. Checking who the manufacturer is and whether or not the expiry date matched with the inner package would also go a long way. Discussing with healthcare providers by any available means and reporting suspicious medicines to the authorities is also very critical. Although measures that are being taken to halt the transmission of COVID-19 are timely and appropriate, it is also highly important to consider the underemployed and the vulnerable segment of the society. They need to be protected both from the pandemic and the consequences of these control measures, consumption of SF medical products in this case. Concerned regulatory bodies shall intervene aggressively in ensuring the safety, quality and effectiveness of medical products before we face a parallel pandemic from SF medical products.
